RETRACTED

# Effect of co-encapsulation using white and red onion peel extract on the viability and stability of *Lacticaseibacillus rhamnosus* under stressful conditions

**DOI:** 10.1371/journal.pone.0311952

**Published:** 2025-03-10

**Authors:** Afaf Ejaz, Yuosra Amer Ali, Muhammad Afzaal, Farhan Saeed, Aftab Ahmed, Sadaf Waliat, Muhammad Umar Farooq, Aasma Asghar, Faiyaz Ahmed, Mahbubur Rahman Khan

**Affiliations:** 1 Department of Food Science, Government College University Faisalabad, Faisalabad, Pakistan; 2 Department of Food Sciences, College of Agriculture and Forestry, University of Mosul, Mosul, Iraq; 3 Department of Nutritional Sciences, Government College University Faisalabad, Faisalabad, Pakistan; 4 Department of Basic Health Sciences, College of Applied Medical Sciences, Qassim University, Buraydah, Saudi Arabia; 5 Department of Food Processing and Preservation, Hajee Mohammad Danesh Science & Technology University, Dinajpur, Bangladesh; NUR International University, PAKISTAN

## Abstract

The study aimed to probe the effect of white and red onion extract on the viability and stability of encapsulated probiotics under stressed conditions. Intentionally, white and red onion peel extract was obtained and used with wall materials to encapsulate the probiotic. Symbiotic microcapsules were characterized for their morphological, molecular, and *in vitro* attributes. Similarly, free and co-encapsulated probiotics cells were also subjected to a simulated gastrointestinal assay. The SEM images demonstrated the successful encapsulation of *Lacticaseibacillus rhamnosus* within sodium alginate, along with white and red onion extract. The FTIR spectra showed the intermolecular interaction between the components of microcapsules. The *in vitro* assay showed that co-encapsulated probiotics showed better survival compared to free cells. In a nutshell, the co-encapsulation with red and white onion extract is an effective approach to enhance the viability of probiotics under stressed conditions.

## 1. Introduction

Probiotics can be co-encapsulated with prebiotics such as polydextrose and inulin to sustain their viability throughout gastrointestinal transit [1]. Antioxidants including tocopherol and ascorbic acid included in microcapsules prevent bacteria from processing and storage-related factors like low pH and oxidative stress [2]. Iyer and Kailasapathy [3] investigated the impact of incorporating resistant starch as a co-encapsulant with chitosan on the viability of probiotics (*Lactobacillus acidophilus* CSSCC 2400 or CSCC 2409). Their findings suggest that hi-maize could significantly enhance the survival of co-encapsulated bacteria, particularly in yogurt or acidic in vitro conditions.

RETRACTED

The onion (*Allium cepa L.*) is ranked as the second most extensively cultivated crop for agricultural purposes globally and holds a significant historical status as one of the oldest and most important vegetable crops known since ancient times. The primary components of onion waste include undersized or defective onions, as well as the outer fleshy layers produced during industrial peeling processes [3]. Proper management of onion waste could be utilized as functional ingredients in the food industry to meet the consumer demands for natural substances over artificial additives. Furthermore, onions constitute a significant dietary reservoir of polyphenols [4]. Onion peel is rich in flavonoids, particularly quercetin and its glycosides, which act as powerful antioxidants and scavengers of free radicals [5]. Additionally, research indicates that onion peel also serves as an important source of inulin and fructooligosaccharides, which are widely recognized as essential prebiotics. Prebiotics are a category of dietary substances that have the ability to promote the growth of specific probiotics, or gut microbiota [6]. The outer layer of onions, known as onion peel has great antioxidant potential with diverse biological properties, presenting potential applications in the pharmaceutical and food industries [7]. Red and white onion varieties contain a substantial amount of phytochemicals, with red onions being especially rich in bioactive constituents such as phenolic acid, organ sulfur compounds, and flavonoids. The peel of onions contains beneficial substances, which have potential protective effects against cardiovascular, cancer, and neurological disorders [8]. In general, red onions contain higher levels of phenolic and flavonoid compounds as compared to white onions [9]. Moreover, approximately 70% of the outer peel of onions consists of a nutritious fiber comprising Microbiota Accessible Carbohydrates (MACs). MACs are carbohydrates that can be utilized by gut microbiota. The purpose of absorbing these carbohydrates is to promote good health. When they traverse through the large intestine without being broken down into smaller pieces in the small intestine, anaerobic bacteria in the large intestine metabolize them to produce organic acids such as butyric, propionic, and acetic acids [10]. These naturally occurring acids play a crucial role in maintaining the balance of intestinal flora in the lower digestive tract [11]. According to Raddatz *et al*. [12] study, red onion peel extracts were successfully added to the micro particles, increasing *Lactobacillus casei* LC03’s probiotic viability in gastrointestinal circumstances. Similarly, probiotic *L. casei* LC03 may be efficiently microencapsulated using 5% extract of red onion peel extract to boost the stability and viability of novel functional foods like strawberry pulp, as reported by Raddatz *et al*. [13] in a different study. The onion peel is a valuable source of functional ingredients. Extracts from both white and red onion peel have the potential to act as prebiotics. It is generally accepted that onion peels are an excellent source of bioactive compounds with antimicrobial and antioxidant properties, including flavonoids and phenolics. However, there has yet to be much research done on their use to enhance the stability of probiotics that have been encapsulated under adverse conditions (such heat, acid, and bile salts). By investigating the potential advantages associated with onion peel extracts on probiotic survival, this investigation seeks to fill this gap. The main objective of this study was to investigate how the extract from two types of onion peel affected the viability and stability of probiotic bacteria when exposed to stressful conditions. Additionally, the study examined the behavior of both free and co-encapsulated probiotics in simulated gastrointestinal conditions.

RETRACTED

## 2. Materials and methods

### 2.1. Materials

The following chemicals were utilized in the current study: sodium alginate, sodium hydroxide, sodium chloride, calcium chloride, and ethanol. These chemicals were all procured from Sigma-Aldrich in the United States and Merck in Germany. The National Institute of Food Science and Technology (NIFSAT) provided probiotic culture (*Lactobacillus. rhamnosus* GG) in freeze-dried form, and the experiment was executed successfully at the Food Safety and Biotechnology Laboratory, Government College University Faisalabad, Pakistan. The experimental design of the study has been showed in Fig 1.

**Fig 1:** Graphical abstract.

### 2.2. Methods

#### 2.2.1. Inoculum preparation.

*Lacticaseibacillus rhamnosus* probiotic culture in freeze-dried condition was anaerobically activated in 100 mL of Man, Rogosa, and Sharpe (MRS) for 20 hours at 37°C. The sample was centrifuged using a Thermo Fisher Scientific 75005286 EA (Thermo Scientific Dionex ICS-5000^+^ Reagent-Free HPIC System) and centrifuge at 6000g for 10 minutes at 4°C. The collected cells were sterilized using 0.85% sodium chloride saline solution, rinsed and place to drt.

#### 2.2.2. Onion peel extraction.

The extracts were obtained using a modified version of the method by Ifesan *et al*. [14]. Initially, the samples were sterilized by using 200 mg/L NaClO (sodium hypochlorite solution) for 20 minutes and then heated in an oven at 50°C for 36 hours. Subsequently, the samples were crushed using a mini mixer grinder. To prepare the extracts, 7 g of red onion peel and 7g of white onion peel were combined with 145 mL of 80% ethanol, respectively. The mixtures were then shaken for four hours at 60°C with a speed of 80 rpm (revolutions per minute). The resulting concentrates were allowed to undergo evaporation, and their volume was adjusted by adding water for subsequent use in various applications [12].

RETRACTED

#### 2.2.3. Microcapsules production by extrusion method.

External ionic gelatin was employed for microencapsulation, as previously reported by de Araújo Etchepare *et al*. [15]. Using extrusion technology, probiotics such as F1, F2, and F3 were encapsulated. F1 contained (2 g/100 mL) sodium alginate particles and *L. rhamnosus*. F2 contained (2 g/100 mL) sodium alginate particles, (2 g/100 mL) red onion peel extract, and *L. rhamnosus*, whereas F3 contained (2 g/100 mL) sodium alginate particles, (2 g/100 mL) white onion peel extract and *L. rhamnosus*. These mixtures were put into an Encapsulator (B-390, Buchi-Switzerland) under standard operating conditions and then each microcapsule was given a unique hardening treatment in 0.1 M CaCl_2_. After whirling the microcapsules in the CaCl_2_ solution for 30 minutes, it was washed with distilled water and the CaCl_2_ was separated using Whatmann filter paper. The obtained beads or microcapsules were collected in polyethylene bags and stored at 4°C to ensure the maximum stability and viability of the encapsulated materials throughout the duration of the experiment or storage period.

### 3.3. Morphological characterization of microcapsules

#### 3.3.1. Size.

The diameters of multiple microscopic particles have been calculated employing a 5 × optical microscope (LABOMED, LX400) [16]. Microcapsules were evaluated shortly after the extraction procedure and under simulated gastrointestinal conditions.

#### 3.3.2. Encapsulation efficiency.

The microcapsules, and efficiency have been examined employing an approach that’s comparable to that stated by Tan and Selig [17]. To determine encapsulation effectiveness, the following computation was applied:


$$EE\left(\%\right)=NE∕\left(NE+Nn\right)\times 100$$

The number of cells not confined (Nn) and the number of cells in microcapsules (NE). The conclusions were shown as CFU/capsule (the general quantity of colonies established).

#### 3.3.3. Zeta potential.

Despite certain modest modifications, by Savadi *et al*. [18] employed to analyze the zeta potential of produced beads. Pure water was employed for the capsules to be dispersed. After distribution, the beads were placed into an experiment sample of a zeta potentiometer (Malvern analytical and Malvern’s Zetasizer Nano ZSP). A period of five minutes was provided for the standard solution to be gradually set. For potential findings, the obtained sample was then placed on a zeta potentiometer.

RETRACTED

#### 3.3.4. Scanning Electron Microscopy (SEM).

The Government College University Faisalabad’s physics department provides an Emcraft Cube II Scanning Electron Microscope (South Korea) with a resolution of 5nm and magnification of up to 200,000x that was utilized to perform scanning electron microscopy on the microcapsules. The specimen’s images were obtained employing a Feld with a working distance of 12.33 mm that was developed in a low vacuum.

### 3.4. Molecular characterization of microcapsules

#### 3.4.1. Fourier Transform Infrared Spectroscopy (FTIR).

FTIR (Fourier transform infrared spectroscopy) is carried out on probiotic-loaded microcapsules employing a method invented by Quan *et al*. [19]. The FTIR methodology was employed together with a Spectroscope “PerkinElmer Spectrum Two FT-IR Spectrometer” (US) available at the National Textile Research Centre NTRC spectroscopy lab at National Textile University Faisalabad to investigate the availability of several functional categories and their impact on the capsules. 30 scans from 550 to 3000 cm^−1^ were utilized at a resolution of 2–3 cm^−1^ for FTIR.

### 3.5. *In vitro* study

#### 3.5.1. Viability of encapsulated *L. rhamnosus* in simulated gastric conditions.

The research conducted by Karim *et al*. [20] checked the probiotic’s viability under simulated gastrointestinal circumstances. Falcon tubes (15 mL) that had undergone sterilization were employed for research. *L. rhamnosus* cells were suspended in 10 mL (0.85%) solution along with pepsin (3 g/L) from Sigma-Aldrich, employing HCL (5M) to encourage gastric conditions pH (2.0). During a period of incubation at 37°C with 70 rpm shaking, 1 mL of samples were discarded at intervals of 0 min, 30 min, 60 min, 90 min, 120 min, and 150 min.

#### 3.5.2. Viability of encapsulated *L. rhamnosus* in simulated intestinal conditions.

To evaluated the probiotic’s performance in simulated gastrointestinal conditions by using the method invented by Shishir *et al*. [21]. Probiotic bacteria’s survival was frequently investigated in a medium that replicated various small intestinal regions. After pH corrections to 5.0 for 20 minutes and to 7.5 for 90 minutes in simulated intestinal condition, *L. rhamnosus* cells were suspended in the pancreas at a concentration of about 2 g L^−1^ (Sigma) and bile salt at a concentration of 12 g L^−1^ of (Sigma). Incubation was carried out in a Daihan Scientific WIS-20 incubating shaker at 150 rpm and 37°C, approximating the temperature of the human body. To find out how long *L. rhamnosus* remained free or encapsulated, the samples were eliminated at intervals of 0 min, 30 min, 60 min, 90 min, 120 min, and 150 min.

RETRACTED

### 2.6. Statistical analysis

The obtained results were reported as the mean ±  standard deviation (SD) of three replicates and were subjected to statistical analysis using a software package for data analysis (SPSS ver. 17.0, SPSS Inc., Chicago, IL, USA). To assess the significance of the differences observed among the means, a one-way analysis of variance (ANOVA) was conducted. The statistical analysis employed Duncan’s test, at a predetermined significance level of 5%.

## 3. Results and discussion

### 3.1. Characterization of microcapsules

#### 3.1.1. Microstructure.

The SEM images presented in Fig 2(a, b) depict the morphological attributes of microcapsules loaded with probiotics. Successful encapsulation of probiotics was confirmed by SEM analysis, revealing their uniform distribution within the microcapsule matrix. The introduction of onion peel extract into the sodium alginate (SA) matrix for *L. rhamnosus* encapsulation yields a notable augmentation in a number of open pores. It was observed that the microcapsules encapsulating *L. rhamnosus* exhibit a slightly rough surface with several pores.

**Fig 2:** Scanning Electron Microscopy (SEM) images of microencapsulated beads with two formulations; sodium alginate and probiotic (a, b), Red onion peel extract with sodium alginate and probiotic (c, d) and White onion peel extract with sodium alginate and probiotic (e, f).

Microcapsules containing probiotics *L. rhamnosus* infused with white onion peel extract exhibited a more textured and heterogeneous surface. Research by Sultana *et al*. [22] indicated that the presence of bacteria and supplementary compounds may impede the proper cross-linking of alginate with calcium chloride, resulting in the final microcapsule product displaying increased porosity. In the present study, SEM demonstrated that introducing onion peel extract decreased the pore size and spherical form of microcapsules because OPE (onion peel extract) comprises fibers and other additives. The microcapsules containing the red onion peel extract were disfigured, shriveled, and rough in appearance see Fig 2(c, d). In comparison to ROPE (red onion peel extract), the WOPE (white onion peel extract) beads showed finer spherical forms. Similar results were observed by Yong *et al*. [23] for the chitosan-based films produced with purple and black rice extracts.

#### 3.1.2. Size, efficiency, and zeta potential of microcapsules.

For SA (sodium alginate), WOPE/SA (white onion peel extract/sodium alginate), and ROPE/SA (red onion peel extract/ sodium alginate), the average microcapsule sizes were 193 ± 0.71 μm, 183 ± 0.56 μm and 181 ± 0.69 μm respectively. These results are consistent with the observations made by de Araújo Etchepare *et al*. [24] who utilized an external ionic gelation approach to fabricate probiotic micro-particles with sizes ranging from 107 to 222 μm.

RETRACTED

Similarly, in another study, Poletto and colleagues employed external ionic gelation followed by freeze-drying to generate micro-particles [25]. These particles exhibited a size range spanning from 127.5 to 234.6 μm. The observed size distribution holds advantageous attributes as it allows any food product to maintain a fine, micrometer-scale smoothness, while concurrently imparting a sandy texture to the product [26]. As concluded in Table 1, it was established that the composition of the wall material exerts a noticeable impact on the dimensions of the micro-particles. In contrast to the conditions involving extract from white onion peel or sole utilization of sodium alginate (SA), the incorporation of the extract from red onion peel led to a notable decrease in the microcapsules’ size from 193 ± 0.71 μm to 181 ± 0.69 μm. It was demonstrated that alterations in the viscosity of the encapsulation solution have the potential to affect the dimensions of the micro-particles [27].

**Table 1:** Characteristics of microparticles containing *L. rhamnosus*, i.e., size, encapsulation efficiency and zeta potential.

Treatment	Size (μm)	Encapsulation Efficiency (%)	Zeta potential (MV)
SA	193 ± 0.71^a^	86 ± 0.69^a^	-14 ± 0.45^a^
ROPE/SA	181 ± 0.69^b^	96 ± 0.33^b^	-38 ± 0.91^b^
WOPE/SA	183 ± 0.56^b^	91 ± 0.49^c^	-35 ± 0.11^bc^

The ±  sign denotes the standard deviations. Row values followed by the letter (a, b, and c) are significantly different (p <  0.05).

Table 1 presents the outcomes derived from assessing the efficacy of probiotic encapsulation within microcapsules both with and without the inclusion of the extract. To ensure the effective delivery of the active component to the desired target site in substantial quantities, the encapsulation methodology must exhibit a notably high degree of retention. The results displayed a notable persistence of probiotics within the capsules (>90%) across all formulations. The addition of onion peel extract to the capsules did not yield any discernible alterations in probiotic proliferation during the encapsulation process. These findings demonstrated that sodium alginate achieved an encapsulation efficiency of 86% for the microcapsules.

The encapsulation efficiency of the microcapsules encapsulated with red onion peel extract 96% was more as compared to 91% of white onion peel extract. This enhancement in effectiveness could be attributed to the heightened bioavailability and solubility of bioactive compounds in red onion peel extract, along with its robust emulsification, gelling, and capacity to generate a highly flexible matrix. According to the study by Thongkaew *et al*. [28] the variation in encapsulation efficiencies between the two extracts could be due to the disruptive impact of polysaccharides on the protein/polyphenol complex within the matrix during the encapsulation process. The findings of the current study are consistent with the previous report [29]. The mean results illustrate the zeta potential values of microcapsules containing sodium alginate and encapsulating two distinct forms of onion peel extract, which are presented in Table 1. The findings showed that the zeta potential of the microcapsules is notably influenced by the nature of the encapsulating materials. For example, the zeta potential value of probiotic *Lacticaseibacillus rhamnosus*, upon encapsulation using sodium alginate, exhibited a measurement of −14 millivolts (mV). However, when encapsulated with a composite of red onion peel extract and sodium alginate, the resulting zeta potential was measured at −38 mV, while utilization of white onion peel extract in conjunction with sodium alginate led to a zeta potential measurement of −35 mV. The zeta potential of probiotics mixed with either variety of onion peel extract exhibited slight differences. Notably, the zeta potential disparity was significantly influenced by the composition of encapsulating materials, the pH of the medium, and the ionic strength. This led to microcapsules demonstrating both positive and negative zeta potential values. These observations highlight the vital role of zeta potential as a determinant of electrochemical properties, as emphasized in reference [30].

RETRACTED

#### 3.1.3. Fourier Transforms Infrared Spectrometry (FTIR).

The molecular makeup of the microcapsules produced through the combination of white and red onion peel extract, sodium alginate, and bacteria was investigated using FTIR analysis (Fig 3(a) and (b)). The specific functional groups are represented by various bonds in the IR spectra. Peaks were observed in the FTIR spectra of the *L. rhamnosus*-containing ROPE/SA microcapsules at 3691 cm^−1^, 2372 cm^−1^, 2335 cm^−1^, 1648 cm^−1^, 1153 cm^−1^, 658 cm^−1^, 636 cm^−1^, 627 cm^−1^ and 625 cm^−1^. The chemical makeup of red onion peel extract microcapsules demonstrated alcohol group by O-H stretching when the medium sharp peak showed up at 3691 cm^−1^ [31]. Two characteristic peaks, one at 2372 cm^−1^ and the other at 2335 cm^−1^, were observed both of which referred to the O=C=O stretching. Previous studies demonstrated a similar FTIR spectrum of the of the onion peel extract with slight differences due to the variations in the concentration [32]. Peaks were evident in the FTIR spectra of the WOPE/SA microcapsules at 2363 cm^−1^, 2335 cm^−1^, 1650 cm^−1^, 781 cm^−1^, 692 cm^−1^, 633 cm^−1^ and 616 cm^−1^. The spectrum showed nearly identical peaks in the case of WOPE/SA mix microcapsules incorporating *L. rhamnosus* as in ROPE/SA. The wavenumbers demonstrated only moderate modifications. In this regard, the peaks at 2372 cm^−1^, and 2335 cm^−1^ in ROPE microcapsules and at 23623 cm^−1^, 2335 cm^−1^ 2372 cm^−1^, and 2335 cm^−1^ in WOPE microcapsules are almost identical. Overall, the FTIR spectra showed intermolecular interaction between the components of the microcapsule [33].

**Fig 3:** The Fourier Transform Infrared Spectroscopy (FTIR) spectra of microcapsules with white onion peel extract, sodium alginate, and probiotic (a) and red onion peel extract with sodium alginate and probiotic (b).

### 3.2. *In vitro* study

#### 3.2.1. Viability and stability of the encapsulated probiotic in simulated gastric conditions.

For probiotics to accomplish their intended impact in gastrointestinal and stomach conditions, the survival of the cells is necessary. The stimulated gastric juice was subjected to both free and encapsulated cells. After preparing synthetic gastric juice (with a pH value of 2.0) and subjecting it to a specific exposure period with a certain period, the stability and viability of free and encapsulated *L. rhamnosus* were examined. Table 2 depicts the overall declining trend in every type of cell that was identified. About encapsulated cells, a sharp decrease in cell number was noted in non-encapsulated cells. From 0 to 60 minutes, the viable probiotic microbial cell count reduced from 8.44 ± 0.05 log CFU/g to 2.18 ± 0.02 CFU/g log in the instance of free cells, suggesting a requirement for protective material. After 60 minutes of assessment, the free cells were not identified in simulated gastric juice (pH 2.0).

**Table 2:** Viability (log CFU/g) of free and encapsulated probiotic bacteria under simulated gastric fluid.

Type of cells	Type of simulated conditions	Time interval (minutes)					
		0 min	30 min	60 min	90 min	120 min	150 min
Free cells	Simulated gastric fluid (pH 2.0)	8.44 ± 0.05^d^	5.87 ± 0.03^j^	2.18 ± 0.02^k^	ND^l^	ND^l^	ND^l^
ROPE/SA blend-loaded probiotics		10.84 ± 0.1^a^	9.78 ± 0.09^b^	8.91 ± 0.03^c^	7.94 ± 0.01^f^	7.42 ± 0.06^g^	7.05 ± 0.17^h^
WOPE/SA blend-loaded probiotics		9.96 ± 0.19^b^	9.08 ± 0.28^c^	8.19 ± 0.31^e^	7.36 ± 0.49^g^	6.53 ± 0.11^i^	6.03 ± 0.07^j^

Data is represented as a mean of triplicate (n = 3). SD is applied ±  at a 5% level of significance.

RETRACTED

The lowercase lettering (a, b, c, etc.) within each row indicates statistically significant differences among the different time intervals for that specific type of cell treatment.

Abbreviation: ND (not detected).

Probiotics cells encapsulated with ROPE/SA, however, demonstrated a drop from 0 to 120 minutes of inspection, falling from 10.84 ± 0.12 log CFU/g to 7.05 ± 0.17 log CFU/g. The total number of probiotic bacterial cells in WOPE/SA encapsulates declined from 9.96 ± 0.19 log CFU/g to 6.03 ± 0.07 log CFU/g. As low pH decreases probiotics’ potential to persist in gastric juice, the viable number of probiotic bacteria in free cells is significantly lowered. Probiotics were no more viable, and no beneficial effects could be achieved.

Probiotics cells enclosed in WOPE/SA, however, exhibited a delayed drop as a result of the encapsulation’s beneficial properties. Results indicated that in comparison to WOPE/SA and free cells, *L. rhamnosus* coated with ROPE/SA demonstrated better stability. This study is in accordance with the findings by Iqbal *et al*. [34] that probiotics sustain longer in stomach environments when they are encapsulated. The findings are also similar to Qi *et al*. [35] who observed that probiotics exhibited a 60% greater viability rate under simulated gastrointestinal conditions compared to free cells (25%), and who ultimately reached the conclusion that probiotics can be efficiently preserved through encapsulation employing biopolymers in detrimental processing and in vitro conditions.

#### 3.2.2. Viability and stability of the encapsulated probiotic in intestinal conditions (pH 7.5).

When subjected to gastrointestinal circumstances, multiple encapsulating substances demonstrate a beneficial influence on probiotics. Free and encapsulated cells were subjected to the synthetic intestine simulation solution for a particular period in the present research. At pH 7.5, a sharp drop in free cells was seen in Table 3 compared to probiotics that were encapsulated. Using either ROPE/SA (red onion peel/sodium alginate) or WOPE/SA (white onion peel/ sodium alginate), *L. rhamnosus* microencapsulation greatly enhanced (p <  0.05). WOPE/SA showed less of an influence than ROPE/SA. From 0 to 90 minutes, the viable probiotic microbial cell count reduced from 8.44 ± 0.06 log CFU/g to 1.05 ± 0.03 log CFU/g, in the instance of free cells, and after 90 minutes of assessment, the free probiotic cells were not identified in simulated gastrointestinal fluid having a pH of 7.5.

RETRACTED

**Table 3:** Viability (log CFU/g) of free and encapsulated probiotic bacteria under simulated intestinal fluid.

Type of cells	Type of simulated conditions	Time interval (minutes)					
		0 min	30 min	60 min	90 min	120 min	150 min
Free cells	Simulated intestinal fluid (Bile salts 0.3%, pH 5.0)	8.44 ± 0.06^g^	5.87 ± 0.04^l^	2.18 ± 0.08^m^	1.05 ± 0.03^n^	ND^o^	ND^o^
ROPE/SA blend-loaded probiotics		10.96 ± 0.0^a^	9.89 ± 0.04^c^	9.09 ± 0.09^e^	8.75 ± 0.01^f^	7.87 ± 0.07^h^	7.55 ± 0.19^i^
WOPE/SA blend-loaded probiotics		10.23 ± 0.0^b^	9.65 ± 0.16^d^	8.84 ± 0.09^f^	7.71 ± 0.11^hi^	6.93 ± 0.21^j^	6.39 ± 0.12^k^

Data is represented as a mean of triplicate (n = 3). SD is applied ±  at a 5% level of significance.

The lowercase lettering (a, b, c, etc.) within each row indicates statistically significant differences among the different time intervals for that specific type of cell treatment.

Abbreviation: ND (not detected).

However, probiotics cells enclosed in ROPE/SA (red onion peel/sodium alginate) revealed a decline after a 120-minute exposure duration ranging from 10.96 ± 0.02 log CFU/g to 7.55 ± 0.19 log CFU/g. The number of probiotic bacterial cells in WOPE/SA (white onion peel/ sodium alginate), encapsulates reduced from 10.04 ± 0.07 log CFU/g to 6.39 ± 0.12 log CFU/g. The probiotic sustainability in simulated intestinal circumstances was boosted by the bioactive substances found within both kinds of onion peel extract and material for walls sodium alginate. Probiotics are influenced by low pH and high pH in both carrier foods and digestive disorders. The current data reflect conclusions that alginate coating promotes discharge and survivability in GIT situations [36]. Researchers have additionally discovered that microparticles can protect the active ingredient in the GI tract while facilitating its dispersion in the ileum [37].

In accordance to these outcomes, co-encapsulation using extracts from the peels of white and red onions may significantly improve *Lacticaseibacillus rhamnosus* viability and equilibrium under stressful conditions, offering a natural and sustainable method for a probiotic encapsulation in the food manufacturing industry. The findings of this study could unlock up the possibility for incorporating naturally occurring antioxidants from food scraps, potentially extending the usefulness and effectiveness of probiotic supplements. The subsequent studies endeavours could concentrate on the optimization of natural extract levels and combination for different strains of probiotics. In execution, this approach can end up in probiotic meals and supplements which are more robust and successful in satisfying consumer demands for organic and health-promoting elements.

RETRACTED

#### 3.2.3. Potential limitations.

**Scalability of the Encapsulation Process:** While the study demonstrates that co-encapsulation using onion peel extracts works effectively in the lab, there could be challenges when encapsulating materials at industrial scale. To make ensure that the method is feasible for commercial use, issues including large-scale production efficiency, uniformity, and cost-effectiveness have to be resolved.

**Variability in Onion Peel Composition:** The bioactive chemical makeup of onion peels may vary significantly depending on onion type, growing circumstances, and processing techniques, among other things. Variability in this respect could affect the consistency of the protective characteristics of the encapsulating material, that could result in differences in probiotic viability and persistence.

#### 3.2.4. Future research directions.

**Optimization of Scaling Techniques:** Further research ought to be focused on developing scalable encapsulation methods that maintain onion peel extracts’ capability to enhance probiotic stability. It would entail developing cutting-edge encapsulation technology and inexpensive techniques for producing excellent encapsulated probiotics on a larger scale.

**Standardization of Onion Peel Extracts:** Additional studies ought to concentrate on regulating the method of extraction to ensure constant levels of bioactive chemicals in order to get around the variation in onion peel composition. It could entail concentrating on specific onion kinds or improving methods of extraction to generate extracts with constant defensive properties.

**Long-term Stability and Shelf-life Studies:** To evaluate the long-term durability and shelf-life of bacteria encapsulated with onion peel extract under different storage conditions, additional research is required. This would yield significant data for the practical application of these encapsulation methods in the food industry.

**Exploration of Other Natural Extracts:** Enhancing upon the findings of this investigation, future research might look into the application of further naturally occurring extracts from food by-products having strong antioxidant and antimicrobial features for probiotic encapsulation, thus broadening the variety of effective natural encapsulating agents that may be employed in the food industry.

## 4. Conclusion

The addition of red and white onion peel extract to encapsulate probiotics is a potential way to extend their survival and stability under stressful conditions. The bioactive compounds and prebiotic potential found in the extract of onion peel help to enhance the viability of probiotics. Compared to free cells, probiotic bacteria that were co-encapsulated with onion peel extract were able to survive better under simulated gastrointestinal conditions. These findings suggest that red onion peel extract is more effective in prolonging the viability of probiotics during technological, gastrointestinal, and processing conditions as compared to white onion peel extract.
